The article "Androgen receptor promotes gastric cancer cell migration and invasion via AKT-phosphorylation dependent upregulation of matrix metalloproteinase 9" was retracted in 2025. Reasons: manipulated images; duplicated images.

# Androgen receptor promotes gastric cancer cell migration and invasion via AKT-phosphorylation dependent upregulation of matrix metalloproteinase 9

**DOI:** 10.18632/oncotarget.2513

**Published:** 2014-09-25

**Authors:** Bao-gui Zhang, Tao Du, Ming-de Zang, Qing Chang, Zhi-yuan Fan, Jian-fang Li, Bei-qin Yu, Li-ping Su, Chen Li, Chao Yan, Qin-long Gu, Zheng-gang Zhu, Min Yan, Bingya Liu

**Affiliations:** ^1^ Shanghai Key Laboratory of Gastric Neoplasms, Department of Surgery, Shanghai Institute of Digestive Surgery, Ruijin Hospital, Shanghai Jiao Tong University School of Medicine, Shanghai, China; ^2^ Department of Surgery, Shanghai East Hospital, Tongji University School of Medicine, No 150 Jimo Road, Shanghai, China

**Keywords:** Androgen receptor, AKT, MMP9, Gastric cancer

## Abstract

Androgen receptor (AR) plays an important role in many kinds of cancers. However, the molecular mechanisms of AR in gastric cancer (GC) are poorly characterized. Here, we investigated the role of AR in GC cell migration, invasion and metastatic potential. Our data showed that AR expression was positively correlated with lymph node metastasis and late TNM stages. These findings were accompanied by activation of AKT and upregulation of matrix metalloproteinase 9 (MMP9). AR overexpression induced increases in GC cell migration, invasion and proliferation *in vitro* and *in vivo*. These effects were attenuated by inhibition of AKT, AR and MMP9. AR overexpression upregulated MMP9 protein levels, whereas this effect was counteracted by AR siRNA. Inhibition of AKT by siRNA or an inhibitor (MK-2206 2HC) decreased AR protein expression in both stably transfected and parental SGC-7901 cells. Luciferase reporter and chromatin immunoprecipitation assays demonstrated that AR bound to the AR-binding sites of the MMP9 promoter. In summary, AR overexpression induced by AKT phosphorylation upregulated MMP9 by binding to its promoter region to promote gastric carcinogenesis. The AKT/AR/MMP9 pathway plays an important role in GC metastasis and may be a novel therapeutic target for GC treatment.

## INTRODUCTION

Gastric cancer (GC), hepatocellular carcinoma (HCC), and pancreatic cancer are all male-predominant cancers [1-3]. In view of this remarkable gender disparity, some studies have explored the importance of the androgen receptor (AR) axis in these cancers [3, 4]. The results have demonstrated that aberrant expression or functions of AR are major contributors to the sex-related disparity in these cancers, which indicated the strong oncogenic properties of AR.

GC is the fourth most common cancer worldwide and more common in developing countries, and the incidence of GC is higher in males than in females with a ratio of 2:1 [1]. Elucidation of the factors causing the sex-related disparity of GC may be important to reveal critical pathways in gastric carcinogenesis. Here, we hypothesized that AR may be responsible for such disparity.

The article "Androgen receptor promotes gastric cancer cell migration and invasion via AKT-phosphorylation dependent upregulation of matrix metalloproteinase 9" was retracted in 2025. Reasons: manipulated images; duplicated images.

AR, also known as NR3C4 (nuclear receptor subfamily 3, group C, member 4), belongs to a family of nuclear receptors that act as transcription factors. Many studies have described the functions of AR in both androgen-dependent and -independent manners [2]. For example, AR overexpression promotes HCC tumorigenicity which may explain the gender disparity of HCC [5, 6]. However, little is known about the mechanism of the disparity in GC. In 1990, Wu demonstrated the presence of AR in GC tissues [7]. Subsequently, some reports have shown the expression of AR in the stomach [8-10]. The significance of AR has been studied for the prognosis of GC, which reported that AR-negative patients show significantly better survival than AR-positive patients. [11]. Besides, An increasing body of evidence from *in vitro* and *in vivo* studies has shown that AR not only mediates the effects of androgen but also functions as an oncoprotein by interacting with other molecules implicating the proliferation and metastasis of cancer cells [12, 13].

Moreover, AR is functionally associated with a broad range of oncogenic signaling pathways. Ha et al found that AR levels are regulated by the AKT [14]. Activation of AKT causes downstream effects such as increases in co-activator binding and chromatin modifications associated with an increase in AR transcriptional output [15]. AKT, also known as protein kinase B, is crucial for regulation of cell proliferation, differentiation, apoptosis, and migration [16, 17]. It is well established that the AKT/P-AKT pathway plays an important role in many kinds of cancers including GC [18, 19].

Recent data have demonstrated that AR is closely related to the development of various types of human cancer by elevating cell migration and invasion in response to various stimuli including inflammatory factors [20]. It is also well known that extracellular matrix (ECM) degradation by matrix metalloproteinases (MMPs) is critical for tumor invasion and metastasis [21]. In GC, MMP2 and MMP9 play an important role in tumor progression, and the degree of MMP2 and MMP9 expression has been shown to correlate with the tumor grade and stage [22]. However, the effect of AR on MMP2 and MMP9 expression in GC is poorly understood.

Here, we investigated AR expression, its relationship to clinicopathological features and P-AKT/MMP9 expression in GC tissues by immunohistochemistry (IHC). Additionally, the effect of AR on the invasion and metastasis of GC cells was examined *in vitro* and *in vivo*. Finally, we characterized the molecular mechanism by which AR mediates the metastatic potential of GC cells.

The article "Androgen receptor promotes gastric cancer cell migration and invasion via AKT-phosphorylation dependent upregulation of matrix metalloproteinase 9" was retracted in 2025. Reasons: manipulated images; duplicated images.

## RESULTS

### AR expression in GC and its correlation with clinicopathological parameters

To explore the role of AR in GC, we performed IHC to analyze the protein expression of 40 GC tissue samples. We identified 15 and 25 GC tissue samples that were positive and negative for AR, respectively. It has been previously reported that dysregulated AR is an independent unfavorable prognostic factor in GC with a positivity rate of 20% [11], the authors' results are in accordance with the reported data (15 out of 40). There was no significant difference between male and female patients in terms of AR expression (positive rate: 10/25 vs 5/15, Table 1). Interestingly, we found a significant difference in the AR positive rate between GC with or without lymph node metastasis (13/25 vs 2/15, Table 1), which has not been described previously. Similarly, we found that the average expression level of AR was significantly upregulated in tumor tissues of patients with later TNM stages (III and V) compared with that in patients with earlier TNM stages (I and II) (14/27 vs 1/13, Table 1). It has also been reported that MMP2 and MMP9 are involved in GC metastasis via the AKT signaling pathway [23]. Therefore, we detected MMP2/MMP9 and P-AKT expression in the corresponding GC tissues using IHC to explore the correlation of AR and some key molecules involved in GC cell migration and invasion. As shown in Table 1 and Fig. 1a, AR expression was positively correlated with the expression of P-AKT and MMP9 but not MMP2. Next, we evaluated the protein expression of AR, P-AKT, MMP2, and MMP9 in the corresponding tissues to validate the results of IHC (Fig. 1b). Collectively, the results provided strong evidence that AR might play a prominent role in gastric carcinogenesis.

**Table 1:** Relationship between AR expression level and clinicopathologic parameters

Clinicopathologic Parameters	Numbers (n)	Positive	Negative	P value
Age (years)				
≤59	18	8	10	N
>59	22	7	15	
Gender				
Male	25	10	15	N
Female	15	5	10	
Bormann Type				
I, II	14	5	9	N
III, IV	26	10	16	
Location				
Middle Proximal	17	6	11	N
Distal	23	9	14	
Diameter (cm)				
≤5	22	8	14	N
>5	18	7	11	
Histologic type				
Intestinal	12	4	8	N
Diffuse	28	11	17	
Depth of invasion				
T1, T2	11	4	7	N
T3, T4	29	11	18	
Lymph node metastasis				
No	15	2	13	0.020
Yes	25	13	12	
Differentiation				
High, Middle	14	5	9	N
Moderate, Low	26	10	16	
TNM stage				
I, II	13	1	12	0.013
III, IV	27	14	13	
P-AKT expression				
Positive	23	12	11	0.046
Negative	17	3	14	
MMP9 expression				
Positive	19	11	8	0.021
Negative	21	4	17	

Abbreviation: N, no significant difference between groups.

The article "Androgen receptor promotes gastric cancer cell migration and invasion via AKT-phosphorylation dependent upregulation of matrix metalloproteinase 9" was retracted in 2025. Reasons: manipulated images; duplicated images.

The AR expression level associated with clinicopathological features, including tumor size, lymph node metastasis, local invasion, and tumor-node-metastasis (TNM) stage are shown. Statistical significance was assessed by Pearson χ2 test.

**Fig.1:** Expression of AR, P-AKT, MMP2, and MMP9 in GC tissues (a) AR, P-AKT, MMP2 and MMP9 protein expression in GC tissues detected by IHC. T2 and T5 were cancer tissues deprived from individuals with or without lymph node metastasis (late or early TNM stage) as shown in Table 1, and they represented cancer tissues with positive and negative expression of AR, respectively. AR, mainly located in nucleus, AKT/P-AKT/MMPs mainly located in cytoplasm and nucleus. (b) Left: AR, P-AKT, MMP2 and MMP9 protein expression in GC tissues detected by WB. Right: densitometric analysis of the bands obtained for each signal. The P-AKT, AR and MMP9 protein levels were higher in T2 than that in T5. Results are expressed as relative expression to control samples. Data are the mean of three independent experiments ± SD (*P<0.05) (original magnification, ×200).

### Overexpression of AR promotes GC cell migration, invasion and proliferation *in vitro*

To elucidate the effect of AR on the malignant phenotypes of GC cells, WB was used to examine the endogenous AR expression of 7 adherent parental gastric cell lines. Our data showed that AR expression level in SGC-7901 cells was lower than CRL-5822 but higher than other cell lines (Fig. 2a), which allowed us to upregulate or downregulate AR conveniently, so we selected it as our tool cell in the following experiments. we assessed the effects of AR overexpression on cell migration, invasion and proliferation, which are key determinants of GC cells. As shown in Fig. 2b, compared with the control, ectopic expression of AR led to significant increases in the migration and invasion of GC cells. The AR overexpression group also showed faster motility in a wound healing assay (P<0.05) (Fig. 2c). Additionally, cells in the AR overexpression group grew more rapidly (Fig. 2d). Taken together, these results indicate a functional role for AR in mediating cell migration, invasion, and proliferation in GC.

**Fig.2:** Effects of AR overexpression on the migration, invasion, and proliferation of SGC-7901 cells (a) Endogenous expression of AR in seven adherent parental GC cell lines. AR expression level in SGC-7901 cells was lower than CRL-5822 but higher than other cell lines. (b) AR promoted the migration and invasion of SGC-7901 cells *in vitro*. Up: Representative photographs of transwell assays. Low: Histograms showed the cell numbers per field of migration (Left) and invasion (Right). (c) Up: Representative photographs of wound healing assays. Low: wound healing curve. AR promoted the wound healing rate of SGC-7901 cells *in vitro*. (d) Cell proliferation curve measured by a Cell Counting Kit-8 assay. Results are the mean of three independent experiments ± SD (*P<0.05) (original magnification, ×200).

The article "Androgen receptor promotes gastric cancer cell migration and invasion via AKT-phosphorylation dependent upregulation of matrix metalloproteinase 9" was retracted in 2025. Reasons: manipulated images; duplicated images.

### AR upregulates MMP9, which depends on the phosphorylation of AKT *in vitro*

As shown in Fig. 1 and Table 1, AR overexpression was accompanied by an increase in the activation of AKT and upregulation of MMP9, which suggests a potential signaling pathway that mediates the effects of AR on gastric carcinogenesis. Molecules involved in the AKT pathway were measured by WB to investigate their distribution. Compared with the control group, we found that the protein expression level of MMP9, but not MMP2, was markedly increased in the AR+ group. In contrast, MMP9 but not P-AKT expression was sharply decreased by AR siRNA (Fig. 3a), which indicate that MMP9 may be in the downstream of the AR. Besides, Compared with the control, when the activity of AKT was blocked by siRNA or the inhibitor, a remarkably decrease in AR expression appeared along with downregulation of MMP9, however, AKT/P-AKT expression was not changed by AR (Fig. 3b and Fig. 3c). Taken together, these data demonstrate that AR upregulates MMP9, which depends on the phosphorylation of AKT.

**Fig.3:** AR upregulates MMP9, which depends on the phosphorylation of AKT *in vitro* (a) Up: AR overexpression upregulated MMP9 (Left). Bar charts represented relative expression of different proteins (Right). Low: AR knockdown by siRNA or inhibitor decreased MMP9 expression. (b) Influence of AKT activity inhibition on endogenous expression of AR. The AR protein level was decreased significantly by siRNA or the inhibitor of AKT, which was accompanied by a decrease in MMP9 expression (Left). Bar charts represented relative expression of different proteins (Right). (c) Effect of AKT inhibition on AR protein expression in stably transfected SGC-7901 cells. AR protein expression was significantly downregulated by inhibition of AKT, which was accompanied by a decrease in MMP9 expression. Results are the mean of three independent experiments ± SD (*P<0.05).

### AR enhances MMP9 expression by binding to its promoter region

As a key transcription factor, AR plays an important role in many pathophysiology processes, including carcinogenesis. To investigate the precise mechanism by which AR promotes the malignant phenotypes of GC, luciferase and chromatin immunoprecipitation (ChIP) assays were performed. We analyzed the MMP9 promoter region for potential AR-binding sites using online tools (http://alggen.lsi.upc.es/cgi-bin/promo_v3/promo/promoinit.cgi?dirDB=TF_8.3 and http://jaspar.genereg.net/), and found two putative sites with high scores (−139 to −148 nt and −1208 to −1223 nt) (Fig. 4a). Then, firefly luciferase reporter plasmids containing the MMP9 promoter with the potential AR-binding sites (MMP9-WT/MT1/MT2) were constructed. Our data showed that the luciferase activity was higher in SGC-7901/AR cells co-transfected with MMP9-WT or MMP9-MT2 than that in control cells. However, the activity was significantly decreased when the cells were transfected with AR-siRNA. Moreover, we found no difference in the luciferase activity between MMP9-MT1 and control groups, which indicate that MT1 might contain the AR-binding site (Fig. 4b). Then the luciferase assay results were validated by ChIP assays (Fig. 4c). Taken together, these data suggest that AR upregulates MMP9 by binding to its promoter.

The article "Androgen receptor promotes gastric cancer cell migration and invasion via AKT-phosphorylation dependent upregulation of matrix metalloproteinase 9" was retracted in 2025. Reasons: manipulated images; duplicated images.

**Fig.4:** AR enhances MMP9 expression by binding to its promoter region in SGC-7901 cells (a) MMP9 promoter region and AR-binding sites predicated by two different on-line tools. Bold on the left indicated the amplified portion of the promoter region, and bold on the right (Up and Low) indicated the binding sites with high scores. (b) Luciferase report assays. A reporter plasmid for MMP9 (pGL3-MMP9) was generated by cloning the MMP9 promoter region (wt) or its mutants (mut1 and mut2) into the pGL3-basic vector. AR significantly increased the luciferase activity of MMP9 promoter region, which was significantly reduced by knockdown of AR. Mut1 may contained the AR-binding site. (c) MMP9 promoter region and AR interaction validated by ChIP assays. MMP9 cDNA was detectable in the immunoprecipitated chromatin samples of SGC7901-AR cells using an antibody against AR, suggesting that AR binds to the MMP9 promoter. Genomic DNA and IgG were used as controls. Results are the mean of three independent experiments ± SD (*P<0.05).

### AR-mediated enhancement of migration, invasion and proliferation can be reversed by inhibition of AR, AKT or MMP9

To examine the effect of AR downregulation on GC cell migration, invasion, and proliferation, we first assessed the effects of AR, AKT and MMP9 inhibition by siRNA or inhibitors on cell motility in wound healing assays. As shown in Fig. 5a, cell motility was decreased significantly after their inhibition, which reversed the differences shown in Fig. 2 (P<0.05). Next, to investigate whether the growth-prompting effect could be reversed by AR or AKT inhibition, AR or AKT was blocked in AR-overexpressing cells followed by analysis of cell proliferation. As a result, the enhancement of proliferation induced by AR was reduced sharply (P<0.05) (Fig. 5b). Then, the migration and invasion of AR-overexpressing cells was assessed after inhibition of AR or AKT or MMP9. As shown in Fig. 5c and Fig. 5d, the data indicated a sharp reversal in the promoting effect of AR on the migration and invasion of SGC-7901 cells (P<0.05). Taken together, these results confirm the functional role of AR in mediating cell migration, invasion and proliferation in GC.

The article "Androgen receptor promotes gastric cancer cell migration and invasion via AKT-phosphorylation dependent upregulation of matrix metalloproteinase 9" was retracted in 2025. Reasons: manipulated images; duplicated images.

**Fig.5:** Effect of AR inhibition on the migration, invasion and proliferation of SGC-7901 cells (a) Enhanced motility of AR-overexpressing cells in the wound healing assay was reversed by inhibition of AR, AKT or MMP9 (Up). Wound healing curve (Low). (b) CCK8 cell proliferation curve. Enhancement of AR-overexpressing cell proliferation was inhibited by suppression of AR or AKT. (c) Transwell assays. The migration-promoting effect induced by AR upregulation was prevented by downregulation of AR or MMP9 or inhibition of AKT *in vitro* (Up). Histograms showed the cell numbers per field of migration (Low). (d) Histograms showed the cell numbers per field of invasion (Up). The invasion-promoting effect induced by AR upregulation was prevented by downregulation of AR, MMP9 or inhibition of AKT *in vitro* (Low). Results are the mean of three independent experiments ± SD (*P<0.05) (original magnification, ×200).

### Overexpression of AR promotes tumor growth and metastasis *in vivo*

We examined whether overexpression of AR could promote tumor growth and peritoneal metastasis *in vivo*. SGC-7901/AR or control cells were injected subcutaneously or peritonealy into nude mice, and subcutaneous tumor formation was monitored by growth curves (Fig. 6a) (P<0.05). After 35 days, the mice were euthanized and subcutaneous tumor weights or peritoneal tumor numbers were assessed. Data indicated that tumors grew slower in the control group than that in the SGC-7901/AR group (Fig. 6a). The average weight of tumors from SGC-7901/AR cells was significantly larger than that of tumors from control cells (2200 ± 190 mg vs. 870 ± 570 mg) (P<0.05). Additionally, as shown in Fig. 6b, the number of tumors of peritoneal metastases in the SGC-7901/AR group was significantly larger than that in the control group (P<0.05).

**Fig.6:** Overexpression of AR promotes tumor growth and migration *in vivo* (a) Photographs of tumors derived from SGC7901/AR and control SGC-7901 cells injected subcutaneously into nude mice. Growth kinetics curve of tumors in nude mice (Low left). Tumor diameters were measured every 7 days. Average tumor weights in nude mice (Low right). AR/Ki-67, mainly located in nucleus, AKT/P-AKT/MMPs mainly located in cytoplasm and nucleus. (b) Photographs of tumors derived from SGC7901/AR and control SGC-7901 cells injected peritonealy into nude mice. The general condition of mice (Up left). Bar charts showed numbers of tumors formed in the peritoneal cavity (Up right). Representative photographs of tumors formed in the peritoneal cavity (Low). (c) Representative IHC photographs of Ki-67 antigen, P-AKT, AR and MMP9 in tumors of nude mice. (d) Representative WB pictures of P-AKT, AR and MMP9 in tumors of nude mice (Left). Bar charts indicated relative expression levels of different proteins (Right). Results are the mean of three independent experiments ± SD (*P < 0.05) (original magnification, ×200).

The article "Androgen receptor promotes gastric cancer cell migration and invasion via AKT-phosphorylation dependent upregulation of matrix metalloproteinase 9" was retracted in 2025. Reasons: manipulated images; duplicated images.

Besides, IHC analysis of Ki-67 antigen revealed that the increased tumor growth in mice was in part owing to more rapid proliferation caused by AR overexpression. The number of Ki-67 antigen-positive cells was higher in tumors derived from SGC-7901/AR cells than that in tumors derived from control cells (P<0.05) (Fig. 6c). To assess whether the correlation between AR and P-AKT or MMP9 could be recapitulated *in vivo*, P-AKT, AR, and MMP9 were detected by IHC (Fig. 6c). The data were consistent with the results in Fig. 1. Next, WB was applied to confirm the results of IHC (Fig. 6d). These data suggest that the promoting effect on tumorigenicity of AR is attributed to increased proliferation and enhanced metastasis *in vivo*.

## DISCUSSION

AR expression has been documented in liver, colon and brain tumors [24-26]. In GC, AR expression has been reported [7] but the precise mechanism by which AR is involved in gastric carcinogenesis has not been explored. Besides, in most studies, it was found to be insignificant or conflicting. Gan et al revealed that AR is expressed independently and shows a decrease in its expression in GC compared with that in adjacent normal tissues [27]. But in a recent study, it was reported that AR-negative patients have significantly better survival than AR-positive patients [11]. The authors' results are in accordance with the reported data that showed AR immunopositivity was observed in 15 out of 40 gastric tumors and its overexpression was positively correlated with lymph node metastasis and late TNM stages. The antibodies employed, sample size, and positive criteria may account for the differences between studies.

The present study revealed that there was no difference in the AR expression of tumors in male and female subjects. This result reflects the fact that activation of the AR pathway can be either ligand dependent or mediated by ligand-independent mechanisms. Castration-resistant prostate cancer may develop as a consequence of the dysregulated AR signaling that results from AR amplifications, altered interactions of co-regulatory molecules during transcription as well as non-steroidal activation by growth factors, cytokines, and neurosecretory products [28].

The article "Androgen receptor promotes gastric cancer cell migration and invasion via AKT-phosphorylation dependent upregulation of matrix metalloproteinase 9" was retracted in 2025. Reasons: manipulated images; duplicated images.

Considering the male predominance of GC and the lack of information available on AR expression in the stomach, detailed mechanistic studies need to be conducted to reveal the mechanism of AR functions in normal stomach and GC. Accumulated evidences implicate AR was involved in the process of carcinogenesis. AR promotes prostate cancer progression by direct suppression of the tumor suppressor gene CCN3/NOV, and it enhances ligand-independent prostate cancer progression through c-Myc upregulation [29, 30]. The aforementioned AR-regulated genes underscore the significance of aberrant AR activity in the development and progression of neoplasia. If we can confirm the role of AR as an important regulator in GC tumorigenicity, AR may serve as a novel prognostic cancer marker and a new target of GC therapeutics.

We demonstrated that AR overexpression promoted GC cell migration, invasion and proliferation, and our results were confirmed by *in vivo* experiments. Recent *in vitro* studies focusing on the molecular interactions of hormone receptors with oncoproteins have been confirmed s in animal models [31, 32]. However, the signaling pathway involved in the AR signal in GC has not been reported. Wang et al indicated that AR can directly interact with PI3 kinase to ultimately upregulate AKT phosphorylation [33]. However, the data are conflicting. Lin et al demonstrated that AR phosphorylation by AKT results in MDM2-mediated ubiquitylation of AR, leading to its proteasomal degradation [34]. These data indicate that the regulation effect of AKT and AR on each other may dependent on the microenviroenment they're involved in, including different co-regulators [35].

Our results indicated that an increase in AKT activity correlated with increased AR protein expression. To confirm this, we assessed the effect of AKT inhibition on GC cells and data showed that AKT suppression resulted in downregulation of AR protein expression and decreases in GC cell migration, invasion, and proliferation. This is the first report to demonstrate that AR induces GC cell migration and invasion via activation of AKT. However, the exact mechanisms by which AR signaling enhanced gastric carcinogenesis remain largely unknown. One potential target by which AR increases the invasion and migration of cancer cells is MMPs. It is well established that secretion of MMPs with the capacity for ECM degradation is a feature of metastatic cancer cells [36]. MMP2 and MMP9 are most well-characterized MMPs with strong proteolytic activity in the ECM [37]. We found that MMP9, but not MMP2, was a key molecule that mediated AKT/AR signals to enhance the metastatic potential of GC, which may be due to different co-regulators that interact with AR in various microenvironments [35]. We also found that the AR-induced upregulation of MMP9 was promoter dependent and these effects were attenuated or inhibited by AR siRNA. Some recent studies have shown that AR upregulates MMP9 expression and activity in prostate cancers [38, 39]. These observations, together with our current findings, may allow us to develop a new therapeutic approach based on targeting these molecules to block GC metastasis.

The article "Androgen receptor promotes gastric cancer cell migration and invasion via AKT-phosphorylation dependent upregulation of matrix metalloproteinase 9" was retracted in 2025. Reasons: manipulated images; duplicated images.

In summary, we have shown for the first time that AR is functionally involved in the regulation of metastasis in GC. This molecular mechanism involves AR-mediated up-regulation of MMP9 via activation of AKT. Our study strongly suggests that the P-AKT/AR/MMP9 pathway may be a potential target for therapeutic strategies to enhance the survival of GC patients.

## METHODS

### Tissues and cell lines

Tissues were resected for GC treatment at Ruijin Hospital, Shanghai Jiao Tong University School of Medicine (Shanghai, China) between 2012 and 2014. Sections were prepared from 10% formalin-fixed, paraffin-embedded GC tissues. All cases of GC were histologically diagnosed according to the Japanese Classification of Gastric Carcinoma and Lauren's classification [40, 41]. Human GC cell lines, SGC-7901, MKN-28, MKN-45, and AGS were purchased from the Shanghai Institutes for Biological Sciences, Chinese Academy of Sciences, and BGC-823 and CRL-5822 GC cell lines were purchased from the American Type Culture Collection (ATCC). The immortalized normal gastric mucosal epithelial cell line GES-1 was a kind gift from Prof. Feng Bin (Sichuan University, Chengdu, China). The cells were cultured routinely in RPMI-1640 supplemented with 10% heat-inactivated fetal bovine serum (FBS), 100U/ml penicillin and 100μg/ml streptomycin in a humidified cell incubator with 5% CO_2_ at 37°C. Exponentially growing cells were used for experiments.

### IHC and WB

For IHC, all staining steps were performed at room temperature and the samples were washed with PBS between steps. Sections were de-waxed before incubation with primary antibodies (rabbit anti-P-AKT/AR/MMP2/MMP9) (Abcam, Cambridge, UK) for 1 h. A biotinylated swine anti-rabbit (Dako, Glostrup, Denmark) secondary antibody was applied for an additional hour following the removal of primary antibodies. Staining was developed with an avidin-biotinylated horseradish peroxidase complex (Dako) and 3, 3′-diaminobenzidine (Dako) following the manufacturer's instructions. Expression of P-AKT/AR/MMP2/MMP9 was detected in the cytoplasm, nuclei or intercellular areas. Positivity of more than 15% of the carcinoma cells was considered as overexpression of the proteins. For WB, tissue samples were lysed using T-PER Tissue Protein Extraction Reagent (Pierce) in the presence of a protease inhibitor cocktail (Pierce). For cultured cells, trypsinized cells were washed with PBS and then subjected to sonication in 50mM Tris-HCl buffer (pH 8.0) containing 1% glycerol, 1mM EDTA, 0.5mM PMSF, and 2mM benzamidine followed by centrifugation. Equal amounts of protein (100μg) were electrophoresed on 12% reducing SDS-polyacrylamide gels. The proteins were electrotransferred to Immobilon-P membranes. The membranes were blocked with 5% non-fat dry milk in Tris-buffered saline (TBS; pH 8.0) containing 0.1% Tween-20 for 2h, and subsequently incubated with rabbit antibodies at 1μg/ml. Antigen-antibody complexes were visualized using enhanced chemiluminescence. In most cases, blots were re-probed with an antibody against glyceraldehyde-3-phosphate dehydrogenase to assess protein loading. Band intensities were quantitated using a Tanon 2500 imaging system (TANON).

The article "Androgen receptor promotes gastric cancer cell migration and invasion via AKT-phosphorylation dependent upregulation of matrix metalloproteinase 9" was retracted in 2025. Reasons: manipulated images; duplicated images.

### Establishment of stable transfectants

Wild-type AR (WT-AR) in a pcDNA3.1 (+) plasmid was kindly provided by Dr. Masahiro Takeyoshi (Research Section I, Chemicals Assessment and Research Center, Chemicals Evaluation and Research Institute, Japan) and Prof. Li-Chun Xu (Xuzhou Medical College). The pcDNA3.1 (+) mammalian expression vector was purchased from NOVOBIO. GC cells were plated at a density of 2 × 10^5^ cells/cm^2^, cultured for 24 h, and then transfected with vectors using 4μg DNA and Lipofectamine (Invitrogen). After 24h, every 48h thereafter for 4 weeks, the culture medium was replaced with fresh medium containing 800μg/ml G418. Pools of 16 clones were isolated as stable transfectants with an AR expression vector or an empty vector.

### Transfection of siRNA and plasmids and inhibitor treatments

SiRNA used in our study mainly target the gene coding regions, which allowed it to knockdown both the endogenous and exogenous AR protein expression effectively and efficiently. 750pmol scrambled siRNA oligos or SiRNAs that specifically targeted human AKT, AR, or MMP9 (Santa Cruz, CA, USA) were transfected into GC cells (2 × 10^6^) using a Lip2000 transfection reagent kit according to the manufacturer's instructions. For plasmid transfections, plasmid DNA and Lipofectamine were diluted separately in serum-free medium and then incubated at room temperature for 5 min. The diluted DNA and Lipofectamine were then mixed and incubated at room temperature for 20 min. Aliquots of the transfection mixture were then added to the cells. For inhibitor treatments, we used an AKT Inhibitor (MK-2206 2HC) (Selleck) at 15nM.

The article "Androgen receptor promotes gastric cancer cell migration and invasion via AKT-phosphorylation dependent upregulation of matrix metalloproteinase 9" was retracted in 2025. Reasons: manipulated images; duplicated images.

### Wound healing assays

GC cells were cultured to 100% confluence in six-well plates. Wound healing assays were performed by scratching the cell monolayer with a sterile 20-μL pipette tip. The cells were then washed once with PBS. Migration of the cells was evaluated at days 1, 3 and 5 under an inverted phase-contrast microscope (Olympus).

### Cell proliferation assays

At 24h post-transfection, cells (2 × 10^3^ cells/well) were seeded into 96-well plates and incubated for 5 days. Cell proliferation was assessed by a water-soluble tetrazolium salt assay using Cell Counting Kit-8 (Dojindo, Kumamoto, Japan) according to the manufacturer's instructions. All experiments were performed in triplicate.

### Cell invasion and migration assays

We employed the Boyden chamber technique (transwell analysis). Briefly, 8μm pore size filters were coated with 100μl of 1mg/ml matrigel (dissolved in serum-free RPMI-1640) (migration assays omit matrigel). A total of 600μl RPMI-1640 containing 10% FBS was added to the lower chambers. Single cell suspensions (1 × 10^5^ cells/well) were added to the upper chambers and allowed to invade for 24h at 37°C in a CO_2_ incubator. Cells remaining attached to the upper surface of the filters were carefully removed with cotton swabs. Invaded cells were stained with 0.1% crystal violet for 10 min at room temperature and examined by light microscopy.

### Luciferase reporter assay

The human MMP9 gene promoter was amplified by PCR and cloned into the multi-cloning site of a pGL3 reporter plasmid (Ambion) containing the WT firefly luciferase reporter gene. To introduce mutations into the seed sequences of the two AR-binding sites in the promoter and generate MMP9 MT1 and MT2 reporters, plasmids were constructed by overlap extension PCR. Cells seeded into 24-well plates were co-transfected with different plasmids (firefly reporter constructs containing the MMP9 promoter, a Renilla-expressing plasmid, pRL-TK, AR plasmid or control plasmid). Firefly and Renilla luciferase activities were measured at 24h post-transfection by the Dual Luciferase Assay System (Promega). Firefly luciferase activity was normalized to Renilla luciferase activity.

### ChIP assay

To evaluate the interaction between AR and MMP9 promoter region, ChIP assays were performed using a kit (Millipore) according to the manufacturer's instructions. Cells were fixed with formaldehyde for protein/DNA crosslinking and then lysed. The DNA was sheared by sonication (15 pulses, 35s on 35s off) and then added to a well coated with an anti-AR antibody. Washes were performed to remove unbound material, and then AR-bound DNA was released by protein digestion with proteinase K. The DNA was purified through a column. PCR was performed using primers designed to target the MMP9 promoter region spanning the site of the interaction with AR. Primers were as follows: MMP9-F: GCAAAGTGTTCATTG GTTAGTGAACTTTAGAACTTCAA; MMP9-R: TTTTTTGCCCCCCACCCCCCGAGAAACAGGGAT TTAAC. Genomic DNA and IgG were used as controls.

The article "Androgen receptor promotes gastric cancer cell migration and invasion via AKT-phosphorylation dependent upregulation of matrix metalloproteinase 9" was retracted in 2025. Reasons: manipulated images; duplicated images.

### *In vivo* experiments

Stably transfected cells with the AR or control plasmid (1 × 10^6^ or 2 × 10^6^ in 150μL) were injected subcutaneously or into the peritoneal cavity of 4-week-old male nude mice (Institute of Zoology, Chinese Academy of Sciences, Shanghai, China). Mice were checked weekly, and tumor nodules were measured with a caliper. Tumor volumes were evaluated using the following formula: volume = (width + length) / 2 × width × length × 0.5236. Mice were sacrificed after 5 weeks. Tumor growth curves and promotion rates were calculated. All tumors were excised, weighed, harvested and embedded in paraffin. A mouse anti-human Ki-67 antigen monoclonal antibody (Dako, 1:50 dilution) was used to determine nuclear expression of Ki-67 by IHC.

### Ethics statement

All animal experiments were conducted according to the Chinese guidelines for animal experimentation and approved by the Institutional Animal Care Committee of Shanghai Jiao-Tong University School of Medicine, Ruijin Hospital. All patients provided written informed consent before enrollment, and the Ethics Committee of Shanghai Jiao-Tong University School of Medicine, Ruijin Hospital approved the study protocol. The study was carried out according to the provisions of the Helsinki Declaration of 1975.

### Statistical methods

Statistical analyses were performed with SPSS Version 19.0 using the Student's t-test or one-way analysis of variance, chi-squared test, Fisher's exact test or Mann–Whitney U-test. Differences were considered statistically significant in two-tailed tests with p-values of <0.05.
